# Combined CNN and Pixel Feature Image for Fatty Liver Ultrasound Image Classification

**DOI:** 10.1155/2022/9385734

**Published:** 2022-12-13

**Authors:** Haijiang Zhu, Yutong Liu, Xiaoyu Gao, Lei Zhang

**Affiliations:** ^1^College of Information & Technology, Beijing University of Chemical Technology, Beijing 100029, China; ^2^Department of Function Test, First Teaching Hospital of Tianjin University of Tradition Chinese Medicine, Tianjin 300193, China

## Abstract

Recent revolutionary results of deep learning indicate the advent of reliable classifiers to perform difficult tasks in medical diagnosis. Fatty liver is a common liver disease, and it is also one of the major challenges people face in disease prevention. It will cause many complications, which need to be found and treated in time. In the field of automatic diagnosis of fatty liver ultrasound images, there are problems of less data amount, and the pathological images of different severity are similar. Therefore, this paper proposes a classification method through combining convolutional neural network with the differential image patches based on pixel-level features for fatty liver ultrasonic images. It can automatically diagnose the ultrasonic images of normal liver, low-grade fatty liver, moderate grade fatty liver, and severe fatty liver. The proposed method not only solves the problem of less data amount but also improves the accuracy of classification. Compared with other deep learning methods and traditional methods, the experimental results show that our method has better accuracy than other classification methods.

## 1. Introduction

Abnormality classification and detection on medical images have attracted the attention of many researchers till the present moment [1–14]. There are the classification of fatty liver disease [1, 4–6], the classification of breast lesions [2, 3, 7, 9, 11, 13], the detection of polycystic ovary syndrome [8], the examinations of the abdominal aorta [10], the brain abnormality classification [12, 14], the lung diseases detection [15, 16], and so on. Researches on classification and detection of medical images are typical for magnetic resonance imaging (MRI), computed tomography (CT), ultrasound image, X-ray image, etc. However, the classification and detection on ultrasound images are more troublesome because of its low contrast and lots of speckle.

Since Hinton and Salakhutdinow [17] have first proposed a deep learning method in 2006, many deep neural networks, such as visual geometry group (VGG) [18], GoogleNet [19], residual network (ResNet) [20], and AlexNet [21], are utilized to medical image classification and detection problems. Maxwell et al. [1] proposed the prediction model for chronic diseases through applying deep learning. Han et al. [2] exploited the deep learning framework to differentiate the distinctive types of lesions and nodules in ultrasound breast images. Shi et al. [3] used stacked deep polynomial network to classify tumor in the breast B-mode ultrasound dataset and prostate ultrasound elastography dataset. Meng et al. [4] investigated a liver fibrosis classification method combining transfer learning (TL) and VGGNet [18]. Talo et al. [12] proposed a deep transfer learning based on ResNet34 model to automatically classify normal and abnormal brain MR images. Xi et al. [13] applied an improved CNN network for automatic feature learning and classifier building on mammography abnormality detection. So far, the number of layers in the reported deep learning networks is several tens of stacked layers (depth) and even up to more than 100 layers. Liu and Fang [22] demonstrated that neural networks with more stacked layers (depth) had not yet shown remarkable advantages compared to conventional methods in a low-level vision task. Therefore, this paper investigated a classification method for fatty liver ultrasonic images using shallow layer CNN.

Fatty liver is an acquired metabolic stress-related liver disorder, and about 20%~30% of the population have fatty liver in China [23]. In general, the texture of the normal liver ultrasonic image is uniform. When fat particles are contained in the liver, the texture of the liver is nonuniform. Thus, pixel-level features play an important role in classification problems for the normal liver images and the fatty liver images. A great deal of computational algorithms, such as gray-level cooccurrence matrix (GLCM) [24, 25], Gabor's filters [26], and wavelet transform [27, 28], has been proposed to analyze the ultrasonic images of the fatty liver in computer-aided diagnosis (CAD) systems. However, there are few researches on classification of fatty liver ultrasound images using deep learning method. Che et al. [29] proposed a multiscale CNN to classify whether there is fatty liver, but this method only studied the binary classification problem and did not classify the degree of disease, similar to [30, 31]. Zamanian et al. [32] proposed the combinational deep learning algorithm, but it combines a variety of network for feature extraction, resulting in a complex network structure.

Due to the particularity of medical imaging, medical images are not as high quality as other natural images, and image annotation can only be performed by professional doctors. In the field of medical image analysis, only a small amount of data can be used to train deep learning models, which often leads to poor results. At the same time, because ultrasound images of fatty liver do not have obvious texture features, it will also lead to CNN difficult to obtain ideal results. As an important factor, statistical regularities of pixel-level features have been utilized for image denoising [22] and hyperspectral image classification-based deep learning [33]. Therefore, in this paper, we combine shallow layer convolutional neural network (CNN) with the differential image patches based on pixel-level features to solve the classification problem of fatty liver ultrasonic images.

The rest of this paper is structured as follows.  Section 2 presents the motive of this work.  Section 3 proposes our convolutional neural network architecture. Experimental results and discussion are given in Section 4, and Section 5 is the conclusions.

## 2. Problem Statement

In a convolutional neural network, the receptive field size of the convolutional filter is enlarged when the networks go deeper. For instance, the geometric receptive size of a stack of two 3 × 3 convolutional layers is equivalent to 5 × 5. Therefore, the features learned by deeper convolutional layers are the abstractions or combinations of the previous features learned by shallower layers. Intuitively, the performance of the networks should improve with the increasing of depth. However, training deep neural networks would be trapped into degradation problems. Such degradation is not caused by overfitting, and adding more layers to a suitably deep model leads to higher training error [20].

The number of features extracted by a convolutional layer is multiplicatively correlated to the width of the network (number of channels). Generally speaking, the widening convolutional networks can help a convolutional layer to learn more features. However, the main features of the liver ultrasonic image are usually the different scale of speckles, whose amount is limited in hundreds. These speckles of the liver ultrasonic image are approximately uniformly distributed. Assuming that, in a 30 × 30 sample image, there are 100 speckles of different shape corresponding to 100 features in the particular layer, the optimal width of this layer is 100. Adding more channels would be just redundant and invalid. Thus, the training performance would not improve continuously with widening the network, but it is saturated.  Figure 1 illustrates the feature maps through the different convolutional layers in the CNN network. From these results, we can see that the texture features of the fatty liver image are obvious after one or three convolutional layers. In addition, the liver texture features are weakened with the convolution layer increases, and this leads to higher training error for a deep model [20].

Inspired by the application of deep learning with pixel-level features [20, 22], this paper first investigates the depth and width of deep learning network for classification of fatty liver ultrasonic images. Then, we propose a classification method through CNN with the differential images based on pixel-level features for the normal liver, low-grade fatty liver, moderate grade fatty liver, and severe fatty liver.

## 3. Our CNN Architecture

The architecture of the proposed network is indicated in Figure 2. It contains two convolutional layers, one pooling layer, and one fully connected layer. Here, we describe data extension strategy based on pixel-level features and determine our network structure components in detail.

### 3.1. Data Extension Strategy Based on Pixel-Level Features

In this section, we propose a data extension strategy for improving the network performance by manipulating its input data. The augmented image data include two parts: original image patches and differential image patches.

In order to train the classifier of fatty liver images, we utilize the ultrasonic image of the normal liver, low-grade fatty liver, moderate grade fatty liver, and severe fatty liver, i.e., 32 images with a 1024 × 768 resolution. About 32 ultrasonic images come from 16 persons which are composed of 4 normal liver, 4 low-grade fatty liver, 4 moderate grade fatty liver, and 4 severe fatty liver. For each ultrasonic image, we use one moving window with the size  *w* to augment the training images.  Figure 3 presents an example of generating image patches through the annotations of the ultrasonic liver images. Each class has about 500 examples, and this amounts to about 2000 training examples.  Figure 4 gives the quantitative and statistical analysis of the training examples of four liver ultrasonic images. The *C*1, *C*2, *C*3, and *C*4 correspond to the normal liver, low-grade fatty liver, moderate grade fatty liver, and severe fatty liver. We can see that most of the image patches have different gray-scale intervals.

From Figure 4, we have found that the gray scale of the fatty liver image *C*1 and *C*2 classes is close, and that of the *C*3 and *C*4 classes is close. Therefore, we propose the image patches expanded strategy based on pixel-level features for the two groups {*C*1, *C*2} and {*C*3, *C*4}.

First, the total average value *ϕ* of the input image patches of *C*1 and *C*2 classes (see Figure 4) is calculated by

(1) $$\begin{array}{c} \phi =\frac{1}{n}\left(\overset{n1}{\underset{i=1}{\sum }}C1_{i}+\overset{n2}{\underset{i=1}{\sum }}C2_{i}\right), \end{array}$$

where *n* = *n*1 + *n*2 is the total number of the image patches in *C*1 and *C*2 classes,  *n*1 is the number of the image patches in *C*1 class, and *n*2 is the number of the image patches in the *C*2 class.

Then, the mean values *φ*_1_ and *φ*_2_ of the image patches in *C*1 class and *C*2 class are estimated from

(2) $$\begin{array}{c} \varphi_{1}=\frac{1}{n1}\overset{n1}{\underset{i=1}{\sum }}C1_{i}, \end{array}$$

(3) $$\begin{array}{c} \varphi_{2}=\frac{1}{n2}\overset{n2}{\underset{i=1}{\sum }}C2_{i}. \end{array}$$

Finally, the differential images DI_*j*_ in *C*1 and *C*2 classes are obtained from

(4) $$\begin{array}{c} {\text{DI}}_{j}={Ι}_{j}-\left(\varphi_{i}-\phi \right),\left(i=1,2;j=1,2,\cdots ,n\right), \end{array}$$

where *Ι*_*j*_ is original image patch.

In this work, we estimated about 250 differential images for *C*1 and *C*2 classes. In order to describe remarkably the differential images based on pixel-level features, the pseudocolor images of the differential images are presented (see in Figure 5). Similarly, the differential images in *C*3 and *C*4 classes are likewise obtained. In a word, we may construct two input data for our CNN architecture, namely, original image patches and differential image patches (see Figure 5).

### 3.2. Determine Structure Components of Our CNN Network

In this section, we investigate an efficient CNN network architecture that can identify four classes of liver ultrasonic images. In order to find the parameters that make the possible optimal performance of our CNN network architecture, we compare the correct identification rate of four classes of liver ultrasonic images on our dataset during training with the different number of layers, different number of filters for each layer, and different filter sizes, respectively.

A CNN is made of three layers: an input layer, multiple hidden layers, and an output layer [21]. The hidden layers typically consist of convolutional layers, pooling layers, fully connected layers, and normalization layers. The convolutional layer is the core of a CNN that carries out most of the computational work. The pooling layer is a form of nonlinear downsampling and may reduce the spatial size of the representation, the number of parameters, and the amount of computation in the network. Fully connected layer is a connection to all activations in the previous layer, and these activations are computed with a matrix multiplication followed by a bias offset. Fan and Farrell [23] demonstrated that deeper network's layers may achieve more powerful the learning capacity in high-level vision tasks. Then, in low-level vision tasks such as pixel-level features, the depth of networks is not the key. Thus, we determine the structure components of our CNN by comparing and analyzing the number of layers, the number of filters, the size of filters, and the normalization layers.

First, we discussed the influence of the different number of layers on the accuracy of the liver image classification. As we can see in Figure 6(a), the performance of CNN is the highest in the liver ultrasonic image classification when the number of the convolutional layer is 2. This result also indicated that fewer network layers might achieve higher performance in low-level vision tasks [5].

Next, the different number of filters in CNNs is implemented to identify the liver ultrasonic images while the number of layers is fixed to 2. We can see that the accuracy of liver images keeps growing vastly in a few training steps while the number of filters is up to 198K from Figure 6(b). These results show that the CNN with 198 K has achieved remarkable performance gains than the networks with other filters 64 K and 250 K.

Third, we analyze the recognition rate of the liver images under the different size of filters when the number of layers and filters is unchanged. From Figure 6(c), we can find that there is almost no difference in the accuracy of three filters with different sizes. However, the filter size of 3 × 3 has a faster convergence speed, and its parameter amount and calculation amount are less than 5 × 5 and 7 × 7. Therefore, the size of final filter is 3 × 3.

Finally, the influence of BN layer to the structure of a neural network is explored. At present, most of the researches on deep learning indicate that adding BN layer may improve the performance of the network. However, is the BN layer necessary in low-level vision tasks [34]? Here, we compare the added BN layer network with the network without BN layer and the result is shown in Figure 6(d). We find that the accuracy of the network with BN layer has very significant fluctuations, and that of the network without BN is more stable.

To summarize, our CNN consists of two convolutional layers, one pooling layer, and one fully connected layer. The number of filters is 198 K, and the size of filter is 3 × 3.

### 3.3. Optimizing the CNN Architecture

In this CNN network, we need to classify four types for all fatty liver images. The output of the network structure is an array, and it contains four elements. Let the output of the fully connected layer be *y*1, *y*2, *y*3, and *y*4; the output is regressed by the softmax function [35].

(5) $$\begin{array}{c} Y\left(i\right)=\text{softmax}\left(y_{i}\right)=\frac{e^{y_{i}}}{\sum_{i=1}^{4}e^{y_{i}}}. \end{array}$$

Obviously, we make the output of each class range from 0 to 1 and ∑_*i*=1_^4^*y*_*i*_ = 1. In our classification model, we aim to learn a mapping function *R*(*i*) = *Y*(*i*; *θ*), where  *θ* is the weight parameter of the network structure. The distance *L*(*θ*) [35] between the true value and the network output is calculated by the cross-entropy function (6). Generally, the smaller the distance, the better the classification effect of the CNN network.

(6) $$\begin{array}{c} L\left(\theta \right)=-\underset{i}{\sum }R\left(i\right)\log Y\left(i;\theta \right), \end{array}$$

where *L*(*θ*) is the loss function. In order to improve the nonlinearity of the proposed network model, we select the rectified linear unit (ReLU) function which is widely used as the activation function. The ReLU function [35] *G*(*h*_*θ*_(*x*)) is written by

(7) $$\begin{array}{c} G\left(h_{\theta }\left(x\right)\right)=\max\left(0,h_{\theta }\left(x\right)\right), \end{array}$$

where *h*_*θ*_(*x*) is the output of the convolutional layers, and *θ* is the weight parameter of the proposed network. When the input is negative, the output of the function becomes zero. This property of ReLU can disable many neurons in the neural network and make the network sparse. This sparsity is very effective for CNN models. In fact, when extracting features, there are not many features in an image. Especially for ultrasonic images of fatty liver, feature information is the most useful information for network models. A large amount of redundant information is not conducive to feature extraction of CNN, improves the training difficulty of the model, and reduces the learning ability. The activation function makes many neural nodes invalid, and it also activates some nodes. The sparse network generated in this way is conducive to more efficient feature extraction of the model.

The network structure is determined by the characteristics of the fatty liver ultrasound image itself. In order to enhance the gray-scale features of fatty liver images, we estimate the difference between different types of images to get the differential image, which can significantly improve the classification accuracy. A skip connection with the differential images is added to the network structure in order to improve the classification accuracy.

In the proposed convolutional network, the characteristics of fatty liver images gradually were reduced with the number of networks increasing because the texture information of the fatty liver images was not very rich. This may lead to a reduction in the accuracy of the classification on fatty liver image. Therefore, we add a skip connection to the proposed network structure. Let *x*_*i*_ be the output of the previous layer and *λ* be a skip connection; the input of the current layer *y*_*i*_ is written by [35]

(8) $$\begin{array}{c} y_{i}=x_{i}+\lambda . \end{array}$$

For the proposed network (see in Figure 1), a skip connection from the input end to the input of the second convolutional layer is added to make up the lost details. In the skip layer, we have sampled the differential images, and the downsampling technology is pooling.

## 4. Experimental Results

### 4.1. Experimental Setting

#### 4.1.1. Training and Testing Data

The fatty liver ultrasound data were obtained from real patients in the hospital with the help of professional radiologists. The image labels are marked by doctors, who judge the image according to clinical experience to determine which type of fatty liver belongs to. For liver ultrasonic images, we choose four types of ultrasonic images: the normal liver, low-grade fatty liver, moderate grade fatty liver, and severe fatty liver. Eight images of size 1024 × 768 pixels were obtained for each class image. And we generated about 500 image patches with same size using the moving windows and about 250 differential images using the data extension strategy based on pixel-level features. This amounts to 3000 training examples, in which each class is equally represented. The image dataset including image patches and the differential images has been divided into a training and a testing set, where the differential images used to build the CNN model are not utilized for the testing set. In the proposed CNN for image classification with known types, we select 50% image patches (1000 patches) and all differential image patches (1000 patches) to train the CNN model and the remaining 50% image patches (1000 patches) for the testing set. The size of the image patches is 28 × 28 pixels.

#### 4.1.2. Parameter Setting and Network Training

All experiments are performed on a computer with an AMD Ryzen 1700 3.0 GHz processor, 16GB of RAM, and GTX 1070Ti graphics cards. We implement the training with step learning rate policy along the basic learning rate of 0.001 and chose Adam as an optimization function. Meantime, the learning rate will gradually decrease with the increase of the epoch.

Through the comparison of the final experimental results, we finally determined that the CNN network structure has two convolution layers, one pooling layer, and one fully connected layer. We used 198 convolution kernels. The parameters in our CNN model are listed in Table 1. The final network structure is not very deep, but very wide, which is more suitable for our fatty liver image.

### 4.2. Comparison with Other Methods

In the first experiment, we compare the proposed CNN adding a skip connection (see the structure of A in Figure 7) with the proposed CNN without a skip connection (see the structure of B in Figure 7). We found that a training network with a deeper structure may cause liver image texture or gray features disappear. The image recognition rate has little improvement with the number of layers increasing. Hence, the differential images are added to the output of the pooling layer in order to avoid the fatty liver image texture or gray features disappear. Figure 7 illustrates the effect of the structure A with a skip connection and the structure B without a skip connection. This result shows that the accuracy of the structure A is higher than that of the structure B after 200 steps of training.

In the second experiment, the proposed CNN method is performed using the image patches with the different size as 28 × 28, 35 × 35, 40 × 40, and 55 × 55 pixels. We can see that there is not much difference between the different size images from Figure 8. The size of 55 × 55 pixels may have higher accuracy in the early stage of training, but its accuracy is decreasing with the number of iterations increasing. This is because the size of the image is too large, and there is an overfitting problem during the iteration. Different size image patches have almost no substantial difference for the accuracy of the image classification. A larger size of 55 × 55 pixels is slightly better in accuracy, but it may have an overfitting problem in training.

The third experiment is that the proposed CNN method is the comparison with several state-of-the-art liver image classification methods, including VGGNet [18], inception-v3 [36], GLCM-svm [24], Gabor's filters-svm [26], and wavelet transform-svm [28].

For the classification of fatty liver images, the most commonly used is GLCM computing eigenvectors to analyze texture features and then classify. Now with the development of deep learning, some networks for image classification have been widely used, such as inception-v3 [36] and VggNet [18]. In this experiment, we classify our experimental datasets using these three networks, and the classification results are listed in Table 2.

From Table 2, VggNet [18] and inception-v3 [36] do not achieve good results for the classification of the fatty liver images although these methods can get a higher recognition rate for natural images. The traditional gray GLCM method [24] also has great limitations for our fatty liver image classification because it is time consuming. The result of wavelet transform [28] is better than that of Gabor's filter [26], but it is inferior to that of the proposed method. Comparing the traditional methods [24, 26, 28], the CNN model can extract deeper features of ultrasound images. At the same time, we compare the complexity of three kinds of networks. The calculation amount corresponds to the time complexity, and the parameter amount corresponds to the space complexity. In the field of deep learning, the indicator commonly used to evaluate the amount of calculation is floating point operations (FLOPs), and the parameter amount is abbreviated as Params. It can be seen that the proposed method has higher FLOPs and Params. This is because this method only uses a small number of layers, which will result in a large shape of the fully connected layer. The fully connected layer produces more than 90% of FLOPs and Params. To sum up, the proposed method uses complexity to exchange precision and has the best results in accuracy and other indicators.

In addition, we also used the networks with the different layers to classify fatty liver images using the same image patches with the size as 40 × 40 pixels. The experimental results are listed in Table 3. We can see that although the network is very deep, the effect is not as good as our shallow network structure. This is because our fatty liver texture features will gradually disappear with the network deepening. When we optimize the use of the jump layer through adding the differential images, the final classification effect is better without increasing the depth of the network structure.

## 5. Conclusion

In this work, we have described a fatty liver image classification method through combining shallow layer convolutional neural network (CNN) with the differential image patches based on pixel-level features. Data extension strategy based on pixel-level features was proposed to augment the dataset of fatty liver ultrasonic images in order to solve the problem of insufficient samples and obscure image texture features. Experimental results show that the proposed method is good enough to boost the accuracy by combining the image patches with differential images of fatty liver ultrasonic images. In the future work, we will continue to study more efficient methods. It is expected to further improve the accuracy and reduce the amount of parameters and calculations. At the same time, we will get a large amount of fatty liver image samples in cooperation with a hospital and will explore the application of this method.

## Figures and Tables

**Figure 1:** The feature maps with the different convolutional layers.

**Figure 2:** The flowchart of the proposed CNN architecture.

**Figure 3:** Example of generating image patches through the annotations of the ultrasonic liver images. (a) An ultrasonic image of normal liver. (b) An ultrasonic image of severe fatty liver. In the normal liver, the echo at the rear of the liver is obvious (marked by five blue arrows in (a)). When a large amount of fat particles is contained in the liver, the liver ultrasonic image turns white and the echo attenuation is serious (marked by two blue arrows in (b)).

**Figure 4:** Quantitative and statistical analysis on the training examples of four liver ultrasonic images. The red line stands for the gray mean, the upper black line is the maximum gray value, and the down black line is minimum gray value.

**Figure 5:** Input windows with  *w* = 28, from original ultrasonic images and differential images. The *C*1, *C*2, *C*3, and *C*4 correspond to the normal liver, low-grade fatty liver, moderate grade fatty liver, and severe fatty liver.

**Figure 6:** Comparison of accuracy on liver ultrasonic images during training for CNNs with different structure components: (a) number of layers, (b) number of filters, (c) size of filters, and (d) with or without BN (batch normalization).

**Figure 7:** Comparison of the accuracy on the structure A with a skip connection and the structure B without a skip connection.

**Figure 8:** Comparison of the accuracy of different sizes.

**Table 1:** The parameters in our CNN model.

1	Input (28 × 28 ultrasound image patches)
2	Conv3: 3 × 3 size, 64 filters, stride = 1, padding = 1
3	ReLU: max (0, *h*_*θ*_(x))
4	Pool: 2 × 2 size, stride = 1
5	Conv3: 3 × 3 size, 198 filters, stride = 1
6	ReLU: max (0, *h*_*θ*_(*x*))
7	FC-19200 (full connect)
8	FC-4 (output of our CNN model)

**Table 2:** The comparison of the proposed method with other three methods.

Methods	Layers	Filters	Filter size	FLOPs (M)	Params (M)	Accuracy	Specificity	Sensitivity
Proposed method	3	198	3 × 3	2448	2376	92%	95%	83%
VggNet [18]	16	512	3 × 3	1055	134	82%	88%	78%
Inception-v3 [36]	22	192	*n* × 1	234	21	85%	90%	79%
GLCM-svm [24]	—	—	—	—	—	79%	81%	46%
Gabor's filters-svm [26]	—	—	—	—	—	54%	55%	46%
Wavelet-svm [28]	—	—	—	—	—	80%	82%	79%

**Table 3:** The comparison of the proposed method with other three methods.

Methods	Filters	Filter size	Accuracy (%)	Specificity	Sensitivity
CNNs with 10 layers (40 × 40) [21]	32	3 × 3	82%	0.88	0.78
CNNs with 20 layers (40 × 40) [21]	32	3 × 3	80%	0.86	0.75
Our CNN without a skip connection	198	3 × 3	88%	0.92	0.81
Our CNN with a skip connection	198	3 × 3	92%	0.95	0.83

## Data Availability

The data used to support the findings of this study were supplied by Professor Zhu under license and so cannot be made freely available. Requests for access to these data should be made to Haijiang Zhu (zhuhj@mail.buct.edu.cn).
